# Identification of Potential miRNA-mRNA Regulatory Network in Denervated Muscular Atrophy by Bioinformatic Analysis

**DOI:** 10.1155/2022/6042591

**Published:** 2022-06-28

**Authors:** Jianhua Wang, Yuhang Liu, Yongming Zhang, Bin Liu, Zhijian Wei

**Affiliations:** ^1^Department of Orthopaedics, Tianjin TEDA Hospital, Tianjin 300457, China; ^2^Department of Orthopaedics, Tianjin Medical University General Hospital, 154 Anshan Road, Heping District, Tianjin, China 300052

## Abstract

Muscle atrophy caused by long-term denervation leads to the loss of skeletal muscle mass and strength, resulting in a poor recovery of functional muscles and decreasing quality of life. Increasing differentially expressed microRNAs (DEMs) have been reported to be involved in the pathogenesis of denervated muscle atrophy. However, there is still insufficient evidence to explain the role of miRNAs and their target genes in skeletal muscle atrophy. Therefore, an integrative exploration of the miRNA-mRNA regulatory network in denervated muscle atrophy is necessary. A total of 21 (16 upregulated and 5 downregulated) DEMs were screened out in the GSE81914 dataset. Med1, Myod1, Nfkb1, Rela, and Camta1 were predicted and verified to be significantly upregulated in denervated muscle atrophy, from which 6 key TF-miRNA relationship pairs, including Med1-mir-1949, Med1-mir-146b, Myod1-mir-29b, Nfkb1-mir-21, Rela-mir-21, and Camta1-mir-132, were obtained. 60 target genes were then predicted by submitting candidate DEMs to the miRNet database. GO and KEGG pathway enrichment analysis showed that target genes of DEMs were mainly enriched in the apoptotic process and PI3K/Akt signaling pathway. Through the PPI network construction, key modules and hub genes were obtained and potentially modulated by mir-29b, mir-132, and mir-133a. According to the qRT-PCR results, the expression of COL1A1 and Ctgf is opposite to their related miRNAs in denervated muscle atrophy. In the study, a potential miRNA-mRNA regulatory network was firstly constructed in denervated muscle atrophy, in which the mir-29b-COL1A1 and mir-133a-Ctgf pathways may provide new insights into the pathogenesis and treatment.

## 1. Introduction

As an important effector organ of the peripheral nervous system, skeletal muscle is controlled and regulated by the peripheral nervous system. Generally, skeletal muscle adapts to slight external changes by secreting myokines and muscle metabolites, thus maintaining the homeostasis of the whole body [1, 2]. Once the peripheral nerve is transected, skeletal muscle is in a state of denervation, which will lead to the loss of signal transmission and material exchange with the peripheral nerve, resulting in a series of pathological changes related to muscular atrophy, including reduction of muscle fiber cross-sectional area and destruction of myofilaments and sarcomere. Skeletal muscle atrophy can lead to poor functional status, reduced quality of life, and adverse impacts on life prognosis in patients, placing a heavy burden on families and society [3, 4]. However, there is no effective treatment strategy for denervated muscle atrophy in clinical practice. Therefore, it is urgent to study the molecular mechanism of muscle atrophy caused by peripheral nerve injury and explore new effective therapeutic targets.

MicroRNAs (miRNAs) are a class of highly conserved regulatory noncoding RNA molecules that consist of 18-25 nucleotides. They can negatively regulate gene expression at the posttranscriptional level by targeting degradation of messenger RNA (mRNA) or blocking protein translation [5, 6]. Studies have shown that dysregulated miRNAs are associated with the occurrence and development of a variety of diseases, including skeletal muscle development and muscle-related diseases. It was reported that many mRNAs play a role in the biological and pathological process of muscle atrophy and regeneration, including mir-1, mir-23a, mir-21, mir-206, and mir-322 [7–9]. In addition, a growing number of studies have used cDNA microarrays to reveal the differential expression of many genes in atrophic muscles. These differentially expressed genes (DEGs) are mainly enriched in biological processes such as activating proteolytic pathways and inhibiting protein synthesis pathways. However, these studies mainly analyze the 7 days (atrophy stage) to 14 days (atrophic fibrosis stage) after sciatic nerve injury. More research on the early stages of denervated muscle atrophy is needed to guide treatment to prevent the progression of the atrophic fibrosis stage [10]. Although many studies have been conducted on the expression and function of miRNA and mRNA in muscle atrophy, few studies have been performed to date on the role of the miRNA-mRNA regulatory network in denervated amyotrophic disease.

In this study, we focused on the early stages of muscle atrophy and screened differentially expressed microRNAs in gastrocnemius muscle after denervation injury 5 days compared with innervation by analyzing a miRNA array. Transcription factors (Tf) and target genes were obtained by predicting DEMs. Then, a functional analysis of target genes was performed to clarify the biological process of muscle atrophy after denervation, and a DEM-hub gene network was conducted to discover key molecular mediators. In addition, the gastrocnemius muscle levels of hub genes were further verified by qQT-PCR. The purpose of this study was to furnish a novel perspective of miRNA–mRNA regulatory network in a model of denervated skeletal muscle atrophy to provide promising targets for denervated muscle atrophy treatment.

## 2. Methods

### 2.1. Animal Experiment

The 6-week-old Sprague-Dawley male rats with the weight of 200 ± 20 g were provided by the Laboratory Animal Center of the Academy of Military Medical Sciences and housed on a 24-hour day-night cycle under temperature 21–23°C. All methods were performed in accordance with the relevant guidelines and regulations.

The animals were randomly divided into experimental group and sham group (*n* = 6 each group). All sciatic nerve transection procedures were standardized and performed under aseptic conditions with the aid of an operating microscope (Motic SMZ171 stereo microscope). For the experimental group, the rats were anesthetized with an intraperitoneal injection of pentobarbital before the sciatic nerve was exposed and cut off through an incision at the mid-thigh region of the hind limb. For the sham group, the rats were operated on a similar surgical procedure but only an incision without sciatic nerve transection. After the operation, all rats received buprenorphine (0.05 mg/kg subcutaneously) to relieve postsurgery pain. Penicillin powder was used on the wounds to prevent infections. The rats were sacrificed by cervical decapitation to harvest gastrocnemius muscle at 5 days postinjury, respectively.

### 2.2. Microarray Analysis and DEM Screening

Downloaded from the GEO database, microRNA profile dataset GSE81914 (Li et al. submitted data 2018) was obtained. GSE81914 is an experimental microarray dataset designed on skeletal muscle atrophy induced by denervation, which includes gastrocnemius muscle samples 5 days after denervation injury (*n* = 4) and sham control (*n* = 4). Its platform is GPL10558 (Affymetrix Multispecies miRNA-3 Array). GEO2R (https://www.ncbi.nlm.nih.gov/geo/geo2r/), an R-based online tool to analyze GEO data [11], was applied to compare and screen DEMs between denervated muscle and innervated muscle. We considered *P* value <0.05 and |logFC|≥1 as the threshold value.

### 2.3. Prediction of Transcription Factors and Target Genes of DEMs

TransmiR is an online transcription factor- (TF-) microRNA (miRNA) regulation database, which has detailed annotations and experimental validation on all TF-miRNA regulations. TransmiR v2.0 database was used to predict the potential upstream transcription factors of candidate DEMs [12]. miRNet is an online tool designed to help elucidate comprehensive microRNA functional annotation, explore miRNAs and their potential targets, and create miRNA-target interaction networks. As a miRNA-centric network visual analytic platform, miRNet was applied to predict the potential downstream target genes of obtained DEMs [13].

### 2.4. Functional Enrichment Analysis

As a database with high data coverage for annotation, visualization, and integrated discovery, DAVID (https://david.ncifcrf.gov/) can provide characteristic gene term enrichment analysis for uploaded gene lists [14]. Gene ontology analysis is widely used to analyze and interpret genomic sequencing because it can annotate genes and gene products [15]. KEGG is a database resource, the desired environment for analyzing variable datasets, containing advanced functional information for understanding gene functions and biological pathways of the cell and the organism [16].

### 2.5. Screening and Analysis of Hub Genes from Integration of PPI Networks

By the Search Tool for the Retrieval of Interacting Genes (STRING), a database widely used to evaluate functional interactions between proteins, we constructed and analyzed the PPI network of target genes. Moreover, we set the comprehensive score >0.4 as the threshold and removed all isolated nodes [17]. Cytoscape software was applied to further visualize and analyze the PPI network. To calculate the number of interconnections and filter highly connected genes, the PPI network was performed by CytoHubba [18]. The top 10 nodes of the PPI network degree score were regarded as hub genes.

### 2.6. qRT-PCR Validation

Total RNA extraction from denervated and innervated gastrocnemius muscle samples with TRIzol Reagent (Invitrogen, USA). Reverse transcriptional PCR was performed to synthesize the complementary DNA (cDNA) by using HiFiScript gDNA Removal RT MasterMix (CWBIO, Beijing, China) following the protocol. The mRNA level was assessed using Universal SYBR Green qPCR Supermix (UE, China) following the instructions. LightCycler® 96 (Roche, China) was applied to conduct real-time PCR, and the relative expression of the candidate gene was calculated by the 2^−*ΔΔ*Ct^ method with the normalization to GAPDH. The sequences of primers are available in Table 1.

### 2.7. Statistical Analysis

All statistical analyses were performed by using IBM SPSS statistic software (version 25.0, Chicago, IL, USA). The results of different groups were represented by the mean ± s.e.m. The comparison of expression levels of denervated and innervated gastrocnemius muscle tissues was analyzed by unpaired, two-tailed Student's *t*-test. *P* < 0.05 was considered to represent a statistically significant difference.

## 3. Results

### 3.1. Identification of DEMs in Denervated Muscle

Based on the analysis of the GSE81914 dataset, the DEM list was obtained with the |logFC| ≥ 1 and *P* value <0.05 as the threshold. Compared with innervated muscle samples, a total of 21 DEMs were detected in denervated muscle samples, including 16 upregulated DEMs and 5 downregulated DEMs. As shown in the volcano plot and cluster heatmap, we extracted a total of 21 DEMs from 1242 miRNAs in the GEO expression matrix and obtained the distribution of upregulated and downregulated DEMs (Figure 1).

### 3.2. Prediction and Validation of Upstream Transcription Factors of DEMs

TransmiR v2.0 database was used to predict the potential upstream transcription factors of candidate DEMs. Of the 21 obtained DEMs submitted to TransmiR v2.0, 11 DEMs were predicted for 14 transcription factors (Figure 2(a)). One transcription factor can act on multiple miRNAs, and one miRNA can also be regulated by more than one transcription factor. For the downregulated DEM, mir-495, the transcription factors were Mlxipl, while for the upregulated DEMs, the transcription factors were Brd4, Hnf4a, Nfkb1, Rela, Gh1, Myod1, Camta1, Mecp2, Nkx2-2, Sox10, Ep300, and Nr3c1. Hnf4a acted on 6 DEMs such as mir-21, mir-132, mir-203, mir-326, mir-511, and mir-1949 simultaneously, while mir-132 was be regulated by 5 transcription factors (Nkx2-2, Mlxipl, Mecp2, Hnf4a, and Camta1).

TF-miRNA regulatory network plays a critical role in regulating denervated muscle atrophy. To obtain the differently expressed transcription factors, we verified the expression trend of transcription factors in the two groups of muscle tissues by qRT-PCR. The results showed that all differently expressed transcription factors, including Med1, Myod1, Nfkb1, Rela, and Camta1, were significantly upregulated in the denervated muscles, which indicated that transcription factors were activated to induce the endogenous expression of a transcriptional program in the pathological process of denervated muscle atrophy (Figure 2(b)). According to the TF-miRNA regulatory network, we identified the key TF-miRNA relationship pairs, including Med1-mir-1949, Med1-mir-146b, Myod1-mir-29b, Nfkb1-mir-21, Rela-mir-21, and Camta1-mir-132.

### 3.3. Prediction and Construction miRNA-mRNA Regulatory Network

Among the candidate DEMs submitted to the miRNet database, a total of 60 target genes were predicted by 11 DEMs, of which 10 upregulated DEMs (mir-29b, mir-21, mir-132, mir-138, mir-203, mir-212, mir-221, mir-222, mir-223, and mir-672) predicted 55 target genes and 1 downregulated DEM (mir-133a) predicted 5 target genes (Table 2). For the 10 upregulated DEMs, mir-29b was identified to potentially target the most genes, with a number of 19. For the 1 downregulated DEM, mir-133a possessed 5 target genes, including Casp9, Ctgf, Hcn2, Klf15, and Slc2a4. For better visualization, we constructed a miRNA-mRNA regulatory network of DEMs and their target genes through Cytoscape software (Figure 3).

### 3.4. GO and KEGG Analysis of Target Genes

To clarify the biological characteristics of target genes related to denervation-induced muscle atrophy, the DAVID was used to perform (Gene Ontology) GO analysis. The obtained results of the enriched GO terms were shown in Figure 4. GO functional enrichment results include gene ontology biological process (BP), molecular function (MF), and cellular components (CC). Our results show that target genes mainly involve biological processes such as cellular response to amino acid stimulus, endodermal cell differentiation, positive regulation of apoptotic process, cell adhesion, cell-matrix adhesion, and cell migration. In the MF group, target genes were mainly enriched in extracellular matrix structural constituent, protein binding, fibronectin binding, protein kinase binding, identical protein binding, kinase binding, and glycoprotein binding. As shown in Figure 4, target genes mainly involve the following cellular components, such as extracellular matrix, collagen trimer, basement membrane, cytosol, collagen type V trimer, cytoplasm, and extracellular space. These data indicated that in the denervation-induced muscle atrophy model, cells in the extracellular matrix, cytoplasm, and collagen trimer perform molecular functions such as protein binding, fibronectin binding, protein kinase binding, and extracellular matrix structural constituent, resulting in cell apoptosis, cell adhesion, and cell migration.

The (Kyoto Encyclopedia of Genes and Genomes) KEGG analysis was applied to explore enriched pathways of target genes. The enriched categories of KEGG pathways are shown in Figure 4(d). Results showed that the PI3K-Akt signaling pathway, protein digestion and absorption, focal adhesion, ECM-receptor interaction, and FoxO signaling pathway were enriched in denervated muscles, which provided molecular pathway mechanisms for studying denervated muscle atrophy.

### 3.5. Module Analysis and Hub Genes Expression Validation

The target genes of denervated gastrocnemius muscle were constructed to construct protein-protein interaction (PPI) networks by using the STRING database. A complex PPI network with 49 nodes and 175 edges was constructed after removing the isolated nodes. Two significant modules with high corresponding degrees, all of which have a score ≥5, were screened by using MCODE in Cytoscape. GO and KEGG enrichment analysis of module 1 and module 2 were displayed in Figure 5. As shown in Figure 5, the target genes of module 1 are regulated by mir-29b and mainly participate in biological processes such as cellular response to amino acid stimulus, endodermal cell differentiation, collagen fibril organization, collagen-activated tyrosine kinase receptor signaling pathway, and cell adhesion. The target genes module 2 are mainly enriched in the biological process of cell apoptosis. The most significant pathway in module 1 and module 2 was simultaneously enriched in the PI3K-Akt signaling pathway.

Among the 49 nodes, there are 18 central nodes that were filtered with the criterion of degree score ≥10. The 18 most crucial genes that shared high interaction were Col1a1, Mmp9, Col4a2, Col3a1, Pten, Col4a1, Mmp2, Col18a1, Col5a2, Vegfa, Ctgf, Foxo3, Col5a1, Col8a1, Col16a1, Col7a1, Col5a3, and Col12a1. Among them, 12 encode collagen-related genes, the target genes of mir-29b, are completely located in module 1(Figure 5(a)). Therefore, we consider that the collagen-related genes regulated by mir-29b play an important role in muscle atrophy. Since COL1A1 has the highest degree value among hub genes and is predominantly expressed in muscle, we selected COL1A1 to represent collagen-related genes for experimental verification. Then, we used qRT-PCR to verify the expression trend of COL1A1, Mmp9, Pten, Mmp2, Vegfa, Ctgf, and Foxo3 (Figure 6). For the upregulated DEM (mir-29b, mir-132, mir-212, and mir-203), unlike the decreased expression of COL1A1, there was no significant change in the expression of Pten, while the expression of Mmp9, Mmp2, FOXO3, and Vegfa increased in contrast. For the downregulated DEM (mir-133a), the expression of Ctgf was significantly increased. Thus, mir-29b-COL1A1 and mir-133a-Ctgf were identified as potential regulatory pathways in denervated muscle.

## 4. Discussion

Due to the slow regeneration of injured axons, it usually takes at least 3 months to regenerate into the distal muscle tissue. After peripheral nerve injury, the target skeletal muscle may result in atrophy by losing its innervation [19, 20]. To improve functional motor recovery, it is necessary to explore the molecular mechanisms and pathological events underlying the progression of denervated muscle atrophy. Nowadays, the development of microarray data technology attracts more and more researchers to obtain a deeper understanding of the related mechanism of denervated skeletal muscle atrophy [21]. In this study, micro-RNA profile dataset GSE81914 was extracted to identify DEMs in the denervated muscle atrophy. Compared with the innervated muscle, a total of 16 upregulated DEMs and 5 downregulated DEMs were differently expressed in the denervated muscle. Among these DEMs, mir-489, mir-381, mir-146b, mir-132, mir-203, mir-21, and mir-29b have been reported to be involved in regulating the pathological process of severe muscle-related diseases, such as cachexia-induced muscle atrophy, immobilization-induced muscle atrophy, aging-induced muscle wasting models, myotonic dystrophy, spinal muscular atrophy, and myopenia [22–26]. However, many miRNAs still need to be further explored in the role of denervated muscle atrophy.

Transcription factors and microRNAs are two significant gene regulatory factors at the transcriptional and posttranscriptional levels. They can mutually regulate one another and form a feed-forward loop to participate in biological processes [27, 28]. Therefore, understanding the crosstalk between the two regulators and their targets is a powerful way to reveal the complex molecular regulatory mechanisms in the denervation-induced muscle atrophy model. Mediator complex subunit 1 (Med1), as a component of the mediator coactivator complex, plays a broad role in nuclear receptor-mediated transcription [29]. In the year 2010, Chen et al. reported that muscle-specific Med1 knockout mice exhibited enhanced insulin sensitivity, improved glucose tolerance, increased mitochondrial density, and promoted the transition of muscles to slow fibers [30]. Overexpression of Med1 inhibits energy expenditure pathways in muscles may be a potential pathway for gastrocnemius atrophy after sciatic nerve transection. Myogenic differentiation 1 (Myod1) acts as a transcriptional activator and promotes the transcription of muscle-specific target genes. It regulates muscle cell differentiation by inducing cell cycle arrest, which is a prerequisite for the initiation of myogenesis. Myod1 has been reported significantly upregulated early after sciatic nerve compression, indicating that it started to play a role in initial muscle atrophy [31]. Studies have shown that mir-29b promotes atrophy of myotubes differentiated from C2C12 or primary myoblasts in vitro and contributes to skeletal muscle atrophy in response to different atrophic stimuli in vivo [26]. Overexpression of myoD resulted in a significant increase in mir-29b levels in L6 cells. Although it has not been verified in vivo [32], these results corroborate our hypothesis that Myod1 may act as a potential regulator of muscle myogenesis by regulating mir-29b expression. RELA protooncogene (Rela), a component of the NF-kappa B complex, and nuclear factor kappa B subunit 1 (Nfkb1) jointly constitute a transcriptionally active NF-kappa B dimer, which participates in the expression of genes in the processes of immunity, inflammation, and apoptosis [33]. Nuclear factor Kappa B (NF-*κ*B) has also been reported to be a prominent signaling molecule in the pathogenesis of skeletal muscle atrophy, and many muscular atrophy-related genes, including MuRF1, MyoD, and cyclin D ubiquitin-binding enzyme (E2), are its target gene [34]. Previous data indicated that NF-*κ*B signaling increased due to aging, and inhibition of p65 reversed muscle atrophy caused by elevated proinflammatory/catabolic cytokines [35, 36]. However, longitudinal studies investigating the role of NF-*κ*B in denervation-induced muscle atrophy are limited. The adverse role of mir-21 has been reported in muscle atrophy following denervation. Moreover, mir-21 has been shown that contribute to muscle fibrosis during Duchenne muscular dystrophy [37]. Furthermore, studies have demonstrated that NF-kappaB mediated mir-21 regulation in cardiomyocyte apoptosis under oxidative stress [38]. CAMTA1 is a member of a family of Ca2+-dependent calmodulin-binding transcription activators conserved in eukaryotes, which encodes protein calmodulin binding transcription activator 1. Previous studies have shown that CAMTA1 was significantly upregulated in stem cells cocultured with the cardiomyocytes system, which enhanced cell-cell communication by inducing Ca (2+) signals, thus activating a myocardial gene program [39]. In addition, Camta1 has been proved to regulate miR-132 to modulate insulin production and secretion in the pathology of the type 2 diabetes rat model [40]. Following that, Med1-mir-1949, Med1-mir-146b, Myod1-mir-29b, Nfkb1-mir-21, Rela-mir-21, and Camta1-mir-132 were predicted to act upstream of neuromuscular process controlling balance. Although in-depth experimental verification is required, we still have evidence to speculate that these key TF-miRNA relationship pairs play an important role in denervated muscle atrophy. In general, these transcription factors also in turn support the importance of these candidate DEMs in the pathogenesis of denervation-induced muscle atrophy.

The GO analysis results showed that the target genes of DEMs in module1 are mainly enriched in biological processes such as collagen fibril organization and cell adhesion, while in module 2, they are mainly enriched in the apoptotic process. In previous studies, activation of apoptotic process in muscle in response to denervation has been amply documented in neuromuscular diseases such as peripheral nerve injury, peripheral neuropathy, and amyotrophic lateral sclerosis (ALS) [41]. A study conducted by Yang et al. showed that denervation drives skeletal muscle atrophy by inducing mitochondrial dysfunction, mitochondrial autophagy, and apoptosis, indicating that inhibiting the apoptotic process is essential before denervated muscle atrophy [42]. Although the changes of collagen fibrous tissue in the process of denervation of muscular atrophy have not been described, Wang et al. have shown that inhibiting microRNA-29 expression promotes collagen expression, which is consistent with our results [43]. KEGG analysis results showed that the target genes of DEMs in the two modules are mainly enriched in the PI3K-Akt signaling pathway. Inactivation of the IGF-1-PI3K-AKT signal will result in increased protein degradation and decreased protein synthesis and will prevent muscle atrophy by inhibiting the FOXO transcription factor. mir-29 has been demonstrated to damage muscle progenitor cell proliferation and induce various types of muscle atrophy by targeting PI3K [26, 44]. In the present study, COL1A1, as a hub target gene of mir-29b, was significantly enriched in collagen fibril organization, extracellular matrix, protein digestion and absorption, and PI3K/Akt signaling pathway. Therefore, mir-29b may regulate the extracellular matrix structural constituent in denervated skeletal muscle by targeting COL1A1 via the PI3K/Akt signaling pathway.

All hub genes in the construction of the DEM-hub gene network were potentially targeted by mir-132, mir-29b, and mir-133a. Among the hub genes verified by qRT-PCR, the expression of Ctgf can constitute a miRNA-mRNA regulatory pathway with mir-133a. mir-133a, a molecular marker for muscle differentiation and atrophy, has become a key regulator of myogenic programs by targeting specific muscle target genes. As a myogenic miRNA, it is involved in the process of muscle remodeling in neuromuscular disorders such as ALS, SMA, and SBMA [45]. However, unlike its expression in other muscle diseases, it decreases in denervated muscles. The expression difference of mir-133a may be regarded as a molecular marker to further elucidate the difference between upper and lower motor neuron neuromuscular diseases. Cell communication network factor 2 (CCN2/CTGF) is well known as a central mediator of tissue remodeling and fibrosis, which can reverse the process of fibrosis by its inhibitory effect. According to reports, CCN2/CTGF levels increase rapidly after skeletal muscle denervation by activating the TGF-*β* signaling pathway [46]. Morales et al. have shown that reducing CCN2/CTGF is beneficial to skeletal muscle and promotes muscle regeneration by reducing fibrosis [47]. The role of mir-133a and Ctgf in the development and regeneration of muscle, and in agreement with the regulatory relationship in the results of this study, indicates that inhibiting the mir-133a-Ctgf pathway may improve denervated muscle atrophy.

Although this is the first analysis to explore the potential miRNA-mRNA regulatory network in denervated muscular atrophy by bioinformatic analysis and qRT-PCR experiments, some limitations of our study need to be considered in depth. Firstly, sufficient sample sizes of different species are needed to further improve the reliability of the analysis. Secondly, we only focused on the miRNA-mRNA regulation relationship in the early stages of denervated muscle atrophy; however, some of these may vary in different stages of denervated muscle atrophy and need more attention. Thirdly, further molecular biological experiments in vivo and in vitro are required to verify the miRNA–mRNA interactions. In addition, due to the limitations of small sample size, a single time point analysis, and a single muscle tissue source, the data analysis of a full-time course, a larger sample size with multiple muscle tissue sources will give us more treatment directions for denervated muscle atrophy.

## 5. Conclusion

In summary, based on the GEO database and bioinformatic analysis, we firstly revealed the regulatory relationship between transcription factors and miRNA and constructed two potential miRNA–mRNA pathways (mir-29b-COL1A1 and mir-133a-Ctgf) in denervated muscle atrophy. Our findings yield new mechanistic insights and molecular targets of effective treatments for denervated muscle atrophy.

## Figures and Tables

**Figure 1:** Identification of the candidate DEMs. (a) Heatmap of the candidate DEMs. Hierarchical clustering heatmap of DEMs screened based on |logFC|≥1 and *P* value <0.05. Color gradient from red to green indicates that the differential gene expression value is from high to low. (b) Volcano plot of DEMs. The *X*-axis is log2 (fold-change) and *Y*-axis is -log10 (*P* value). Red points (fold change >2) indicate upregulated miRNAs and blue points (fold change <-2) indicate downregulated miRNAs. The black points represent genes with no significant difference.

**Figure 2:** Potential transcription factors of DEMs. (a) Potential tf-miRNA regulatory network predicted and constructed by TransmiR. (b) qRT–PCR analysis showed Hnf4a, Nkx2-2, Mlxipl, and Med1 expressions in gastrocnemius muscle from denervation rats compared to controls. Error bars, s.e.m. An unpaired, two-tailed Student's *t*-test was used for comparisons between the two groups. ^∗^*P* < 0.05, ^∗∗^*P* < 0.01, and ^∗∗∗^*P* < 0.001.

**Figure 3:** Potential target genes of DEMs predicted by miRNet.

**Figure 4:** The GO enrichment and KEGG pathway analysis of the target genes. (a)–(c) The top 10 GO enrichment terms of the target genes based on biological processes (BP), cell compositions (CC), and molecular functions (MF). (d) The top 10 KEGG pathways analysis terms of the target genes. The three parameters of gene ratio, gene count, and -log10 (*P* value) were used to evaluate enrichment items.

**Figure 5:** Construction of PPI and module analysis. (a) The first module and nodes. (b) The enrichment GO term of module 1. (c) The second module and nodes. (d) The enrichment GO term of module 2.

**Figure 6:** Identification and validation of hub gene expression. (a) PPI network of the top 18 hub genes. (b) The mRNA expression of the hub genes was validated by qRT–PCR. Error bars, s.e.m. An unpaired, two-tailed Student's *t*-test was used for comparisons between the two groups. ^∗^*P* < 0.05, ^∗∗^*P* < 0.01, and ^∗∗∗^*P* < 0.001.

**Table 1:** Primer sequences.

Gene	Forward primer sequence (5′-3′)	Reward primer sequence (5′-3′)
Col1a1 Mmp9	GGGTCTAGACATGTTCAGCTTTG CCACTAAAGGTCGCTCGGAT	GGCAGTGGCCCCTAAGAG GAGTTGCCCCCAGTTACAGT
Pten	CATGAGCGAGTTGGTCAAGA	CCATGCTGTGCTGGTTCA
Mmp2	GCACCGTCGCCCATCA	GCACTGCCAACTCTTTGTCTGTT
Vegfa	CGA AAC CAT GAA CTT TCT GC	CCT CAG TGG GCA CAC ACT CC
Ctgf	CAGGGAGTAAGGGACACGA	ACAGCAGTTAGGAACCCAGAT
FOXO3	GCTAAGCAGGCCTCATCTCA	TTCGGTCAGTTTGAGGGTCT
Hnf4a	TGCCAACCTCAACTCATCCAACAG	TCCTCACGCTCCTCCTGAAGAATC
Mlxipl	CGACACTCACCCGCCTCTTC	TTGTTCAGCCGAATCTTGTC
Med1	AGGAGAAGCGGCAGGATAAAC	GTACACGTTGACTTCATGTCCTT
Nkx2-2	TCTACGACAGCAGCGACAAC	CTTGGAGCTTGAGTCCTGAG
Myod1	CCCTGTTGTTTGTGGAGACA	CTGTGGGAAAGAGTGGGTGT
Nfkb1	TTCCTGATCCCGACAAGAACTG	CCCCCAGAGACCTCATAGTTGT
Rela	CCATCAGGGCAGATCTCAAACC	GCTGCTGAAACTCTGAGTTGTC
Nr3c1	CTTGAGAAACTTACACCTCGATGACC	AGCAGTAGGTAAGGAGATTCTCAACC
Camta1	CTGGGAGATGACCTTCACG	GGACAAGCTCCCCATCACAG
Mecp2	CAGCTCCAACAGGATTCCATGGT	AGGCAGGCAAAGCAGAGACATCA
Ep300	AAAAATAAGAGCAGCCTGAG	AGACCTCTTTATGCTTCTTCC
Sox10	ATCCAGGCCCACTACAAGAGC	ATGTCCACGTTGCCGAAGT
Gh1	CATGCCCTTGTCCAGTCTGT	AATGTAGGCACGCTCGAACT
Brd4	TGAGCAGATATTGCAGTTGGTT	CCTCCCAAATGTCTACAACGC
GAPDH	GACATGCCGCCTGGA GAAAC	AGCCCAGGATGCCCTTTAGT

**Table 2:** Potential target genes of the DEMs.

DEMs	Expression	Count	Target genes
mir-132	Up	10	Arhgap32, Capn8, Cyp2e1, Foxo3, Grin2a, Lrrfip1, Mecp2, Mmp9, Pten, Rasa1
mir-133a	Down	5	Casp9, Ctgf, Hcn2, Klf15, Slc2a4
mir-138	Up	3	Lypla1, Rhoc, Vim
mir-203	Up	2	Trpv4, Vegfa
mir-21	Up	15	Capn8, Elavl4, Faslg, Kcnj16, Nqo1, Pdcd4, Pdpn, Peli1, Pten, Rad23, Rela, RGD1565591, Tagln, Tiam1, Tpm1
mir-212	Up	4	Cyp2e1, Foxo3, Pten, Rasa1
mir-221	Up	3	Bcl2l11, Cdkn1b, Cdkn1c
mir-222	Up	3	Bcl2l11, Cdkn1b, Cdkn1c
mir-223	Up	4	Aqp4, Cntn4, Scn3a, Vim
mir-29b	Up	19	Cav2, Col12a1, Col16a1, Col18a1, Col1a1, Col3a1, Col4a1, Col4a2, Col5a1, Col5a2, Col5a3, Col7a1, Col8a1, Dnmt3b, Insig1, Itgb1, Mmp2, Stx1a, Vegfa
mir-672	Up	2	Fndc1, Tnfsf10

## Data Availability

The datasets generated and analyzed during the current study are available in GEO (http://www.ncbi.nlm.nih.gov/geo/).

## Abbreviations

DEM: Differentially expressed microRNA
DEG: Differentially expressed gene
miRNA: MicroRNA
mRNA: Messenger RNA
TF: Transcription factor
GO: Gene Ontology
KEGG: Kyoto Encyclopedia of Genes and Genomes
BP: Biological process
MF: Molecular function
CC: Cellular components
PPI: Protein-protein interaction.

## Additional Points

*Preprint Statement*. A preprint has previously been published and is available from https://www.researchsquare.com/article/rs-864617/v3.

## References

[1] Aversa Z., Zhang X., Fielding R. A., Lanza I., LeBrasseur N. K. (2019). The clinical impact and biological mechanisms of skeletal muscle aging. *Bone*.

[2] Midrio M. (2006). The denervated muscle: facts and hypotheses. A historical review. *European journal of applied physiology*.

[3] Reza M. M., Subramaniyam N., Sim C. M. (2017). Irisin is a pro-myogenic factor that induces skeletal muscle hypertrophy and rescues denervation-induced atrophy. *Nature Communications*.

[4] Gu X., Ding F., Yang Y., Liu J. (2011). Construction of tissue engineered nerve grafts and their application in peripheral nerve regeneration. *Progress in Neurobiology*.

[5] Ivey K. N., Srivastava D. (2015). MicroRNAs as developmental regulators. *Cold Spring Harbor Perspectives in Biology*.

[6] Bartel D. P. (2009). MicroRNAs: target recognition and regulatory functions. *Cell*.

[7] Wada S., Kato Y., Okutsu M. (2011). Translational suppression of atrophic regulators by microRNA-23a integrates resistance to skeletal muscle atrophy. *The Journal of Biological Chemistry*.

[8] Kukreti H., Amuthavalli K., Harikumar A. (2013). Muscle-specific microRNA1 (miR1) targets heat shock protein 70 (HSP70) during dexamethasone-mediated atrophy. *The Journal of Biological Chemistry*.

[9] Soares R. J., Cagnin S., Chemello F. (2014). Involvement of microRNAs in the regulation of muscle wasting during catabolic conditions. *The Journal of Biological Chemistry*.

[10] Shen Y., Zhang R., Xu L. (2019). Microarray analysis of gene expression provides new insights into denervation-induced skeletal muscle atrophy. *Microarray Analysis of Gene Expression Provides New Insights Into Denervation-Induced Skeletal Muscle Atrophy.*.

[11] Barrett T., Wilhite S. E., Ledoux P. (2013). NCBI GEO: archive for functional genomics data sets--update. *Nucleic Acids Research*.

[12] Tong Z., Cui Q., Wang J., Zhou Y. (2019). TransmiR v2.0: an updated transcription factor-microRNA regulation database. *Nucleic Acids Research*.

[13] Chang L., Zhou G., Soufan O., Xia J. (2020). miRNet 2.0: network-based visual analytics for miRNA functional analysis and systems biology. *Nucleic Acids Research*.

[14] Huang D. W., Sherman B. T., Tan Q. (2007). DAVID Bioinformatics Resources: expanded annotation database and novel algorithms to better extract biology from large gene lists. *Nucleic acids research*.

[15] Botstein D., Cherry J. M., Ashburner M. (2000). Gene Ontology: tool for the unification of biology. *Nat genet*.

[16] Altermann E., Klaenhammer T. R. (2005). PathwayVoyager: pathway mapping using the Kyoto Encyclopedia of Genes and Genomes (KEGG) database. *BMC Genomics*.

[17] Franceschini A., Szklarczyk D., Frankild S. (2013). STRING v9.1: protein-protein interaction networks, with increased coverage and integration. *Nucleic Acids Research*.

[18] Chin C. H., Chen S. H., Wu H. H., Ho C. W., Ko M. T., Lin C. Y. (2014). cytoHubba: identifying hub objects and sub-networks from complex interactome. *BMC Systems Biology*.

[19] Höke A., Brushart T. (2010). Introduction to special issue: challenges and opportunities for regeneration in the peripheral nervous system. *Experimental Neurology*.

[20] Weng J., Zhang P., Yin X., Jiang B. (2018). The whole transcriptome involved in denervated muscle atrophy following peripheral nerve injury. *Frontiers in Molecular Neuroscience*.

[21] Li G., Li Q. S., Li W. B. (2016). miRNA targeted signaling pathway in the early stage of denervated fast and slow muscle atrophy. *Neural Regeneration Research*.

[22] Moraes L. N., Fernandez G. J., Vechetti-Júnior I. J. (2017). Integration of miRNA and mRNA expression profiles reveals microRNA-regulated networks during muscle wasting in cardiac cachexia. *Scientific Reports*.

[23] Greco S., Perfetti A., Fasanaro P. (2012). Deregulated microRNAs in myotonic dystrophy type 2. *PLoS One*.

[24] Catapano F., Zaharieva I., Scoto M. (2016). Altered levels of microRNA-9, -206, and -132 in spinal muscular atrophy and their response to antisense oligonucleotide therapy. *Molecular therapy. Nucleic acids*.

[25] Okugawa Y., Toiyama Y., Hur K. (2019). Circulating miR-203 derived from metastatic tissues promotes myopenia in colorectal cancer patients. *Journal of Cachexia, Sarcopenia and Muscle*.

[26] Li J., Chan M. C., Yu Y. (2017). miR-29b contributes to multiple types of muscle atrophy. *Nature Communications*.

[27] Xie G.-Y., Xia M., Miao Y. R., Luo M., Zhang Q., Guo A. Y. (2020). FFLtool: a web server for transcription factor and miRNA feed forward loop analysis in human. *Bioinformatics (Oxford, England)*.

[28] Hobert O. (2008). Gene regulation by transcription factors and microRNAs. *Science (New York, N.Y.)*.

[29] Belakavadi M., Fondell J. D. (2006). Role of the mediator complex in nuclear hormone receptor signaling. *Reviews of Physiology, Biochemistry and Pharmacology*.

[30] Chen W., Zhang X., Birsoy K., Roeder R. G. (2010). A muscle-specific knockout implicates nuclear receptor coactivator MED1 in the regulation of glucose and energy metabolism. *Proceedings of the National Academy of Sciences of the United States of America*.

[31] Grönholdt-Klein M., Altun M., Becklén M. (2019). Muscle atrophy and regeneration associated with behavioural loss and recovery of function after sciatic nerve crush. *Acta Physiologica (Oxford, England)*.

[32] Liu C. Z., Li J. J., Su J. M. (2013). Expression of microRNA-29b2-c cluster is positively regulated by MYOD in L6 cells. *Chinese Medical Sciences Journal*.

[33] Cai D., Frantz J. D., Tawa N. E. (2004). IKK*β*/NF-*κ*B activation causes severe muscle wasting in mice. *Cell*.

[34] Pahl H. L. (1999). Activators and target genes of Rel/NF-*κ*B transcription factors. *Oncogene*.

[35] Buford T. W., Cooke M. B., Manini T. M., Leeuwenburgh C., Willoughby D. S. (2010). Effects of age and sedentary lifestyle on skeletal muscle NF- B signaling in men. *The Journals of Gerontology. Series A, Biological Sciences and Medical Sciences*.

[36] Yamaki T., Wu C. L., Gustin M., Lim J., Jackman R. W., Kandarian S. C. (2012). Rel A/p65 is required for cytokine-induced myotube atrophy. *American Journal of Physiology. Cell Physiology*.

[37] Borja-Gonzalez M., Casas-Martinez J. C., McDonagh B., Goljanek-Whysall K. (2020). Inflamma-MiR-21 negatively regulates myogenesis during ageing. *Antioxidants*.

[38] Wei C., Li L., Kim I. K., Sun P., Gupta S. (2014). NF-*κ*B mediated miR-21 regulation in cardiomyocytes apoptosis under oxidative stress. *Free Radical Research*.

[39] Muller-Borer B., Esch G., Aldina R. (2012). Calcium dependent CAMTA1 in adult stem cell commitment to a myocardial lineage. *PLoS One*.

[40] Mollet I. G., Malm H. A., Wendt A., Orho-Melander M., Eliasson L. (2016). Integrator of stress responses calmodulin binding transcription activator 1 (Camta1) regulates miR-212/miR-132 expression and insulin secretion. *The Journal of Biological Chemistry*.

[41] Siu P. M. (2009). Muscle apoptotic response to denervation, disuse, and aging. *Medicine and Science in Sports and Exercise*.

[42] Yang X., Xue P., Chen H. (2020). Denervation drives skeletal muscle atrophy and induces mitochondrial dysfunction, mitophagy and apoptosis via miR-142a-5p/MFN1 axis. *Theranostics*.

[43] Wang B., Komers R., Carew R. (2012). Suppression of microRNA-29 expression by TGF-*β*1 promotes collagen expression and renal fibrosis. *Journal of the American Society of Nephrology : JASN*.

[44] Hu Z., Klein J. D., Mitch W. E., Zhang L., Martinez I., Wang X. H. (2014). MicroRNA-29 induces cellular senescence in aging muscle through multiple signaling pathways. *Aging*.

[45] Malacarne C., Galbiati M., Giagnorio E. (2021). Dysregulation of muscle-specific microRNAs as common pathogenic feature associated with muscle atrophy in ALS, SMA and SBMA: evidence from animal models and human patients. *International Journal of Molecular Sciences*.

[46] Rebolledo D. L., González D., Faundez-Contreras J. (2019). Denervation-induced skeletal muscle fibrosis is mediated by CTGF/CCN2 independently of TGF-*β*. *Matrix biology : journal of the International Society for Matrix Biology*.

[47] Morales M. G., Gutierrez J., Cabello-Verrugio C. (2013). Reducing CTGF/CCN2 slows down mdx muscle dystrophy and improves cell therapy. *Human Molecular Genetics*.

